# Effect of Percutaneous Nephrolithotomy Combined with Needle Nephrolithotomy on Renal Function and Complication Rate in Patients with Complex Renal Calculi

**DOI:** 10.1155/2022/7312960

**Published:** 2022-09-19

**Authors:** Guangcheng Ge, Chenghao Wang

**Affiliations:** Zhenjiang Hospital of Chinese Traditional and Western Medicine Urology Surgery, Zhenjiang 212000, China

## Abstract

**Objective:**

To investigate the effect of percutaneous nephrolithotomy combined with needle nephrolithotomy on renal function and incidence of complications in patients with complex renal calculi.

**Methods:**

From March 2020 to March 2022, 88 patients with complex renal calculi were enrolled and divided into two groups. Percutaneous nephrolithotomy (PCNL) was performed in the control group, and percutaneous nephrolithotomy combined with needle nephrolithotomy was performed in the study group. Perioperative conditions, renal function parameters such as blood urea nitrogen (BUN), serum creatinine (Scr), and cystatin C (CysC) levels, inflammatory factors such as C-reactive protein (CRP) and procalcitonin (PCT) levels before surgery and 1 day after surgery were determined. The incidence of complications was statistically analyzed between two groups.

**Results:**

There was no significant difference in stone clearance rate between the two groups. The operation time and hospital stay in the study group were shorter than those in the control group. The intraoperative blood loss was less than that in the control group. The VAS score was lower than that in the control group. BUN, Scr, and CysC in the study group were not significantly different from those in the control group. CRP and PCT in the two groups at 1 d after surgery were higher than those before surgery, but CRP and PCT in the study group were lower than those in the control group. The incidence of complications in the study group was lower than that in the control group.

**Conclusion:**

Percutaneous nephrolithotomy combined with needle nephrolithotomy is effective and safe in the treatment of complex renal calculi.

## 1. Introduction

The incidence of kidney stones is high. Complex kidney stones are mainly staghorn-shaped or multiple and large stones with a diameter of ≥2.5 cm. In general, stones are numerous, widely distributed, and difficult to remove, posing a great threat to the quality of life and physical and mental health of patients [1, 2]. Therefore, timely, safe, and effective treatment for patients with complex kidney stones is of great significance. Surgery is an important treatment for complex kidney stones. Traditional open surgery is more traumatic and has a higher incidence of postoperative complications, which gradually makes it difficult to meet the actual clinical needs [3–5]. Percutaneous nephrolithotomy (PCNL) is also an important treatment for complex kidney stones. Compared with laparotomy, PCNL has less trauma and faster recovery of physical function after surgery, but there may still be related complications such as organ damage, infection, and bleeding after surgery [6–8]. Needle nephroscope is a new type of PCNL device, which mainly includes a needle handle and a puncture outer sheath. The tail of the needle handle is a three-way device, which can be connected to a titanium laser fiber (200 *μ*m), a video introduction fiber, and a liquid perfusion device, which is of great significance for improving the efficacy and safety of the treatment [9]. Based on this, this study planned to select 88 patients with complex renal calculi in our hospital, and grouped to explore the intervention value of percutaneous nephrolithotomy combined with needle nephrolithotomy.

## 2. Materials and Methods

### 2.1. General Information

Eighty-eight patients with complex renal calculi in our hospital from March 2020 to March 2022 were enrolled. The inclusion criteria were as follows: (1) confirmed by CT, urography, and transabdominal ultrasonography; (2) multiple or calculi with long diameter ≥2.5 cm and surface area >500 mm^2^; (3) aware of this study and signed the consent form; and (4) single renal calculi. The exclusion criteria of this study were as follows: (1) Patients with coagulation disorders; (2) Patients with diabetes, hypertension, and chronic nephritis; (3) Patients with immune system diseases; (4) Patients with malignant tumors; (5) Patients with a history of surgical treatment of urinary calculi; (6) Lactating and pregnant women. They were divided into the study group and the control group according to simple random number table, 44 cases for each group. The study group consisted of 26 males and 18 females, aged 34∼69 years, with mean one of (51.38 ± 12.71) years; affected side: left kidney in 27 cases, right kidney in 17 cases; stone type: multiple in 22 cases, cast in 16 cases, staghorn in 6 cases. The control group consisted of 28 males and 16 females, aged 32∼69 years, with mean one of (50.81 ± 14.04) years; affected side: 25 cases of left kidney and 19 cases of right kidney; stone types: multiple in 18 cases, cast in 18 cases, and staghorn in 8 cases. There were no significant differences in clinical data between two groups (*P* > 0.05). The protocol of this study was approved by the Ethics Committee of Zhenjiang Hospital of Chinese Traditional and Western Medicine Urology Surgery.

### 2.2. Treatment

For the patients in the control group, PCNL was adopted, general anesthesia was given, lithotomy position was taken, the ureterorenoscope (F9.8) was inserted into the F5 ureteral catheter through the bladder, it was inserted into the renal pelvis, the ureteral catheter was properly fixed, an appropriate amount of normal saline was injected for those without hydronephrosis, abdominal pad height, the renal condition was identified, the puncture point was selected, puncture treatment through the puncture needle (18 G) of the target calyx was performed, incise the skin at the puncture site, the fascial dilator was placed, it was dilated to 16 F, F 18 soft sheath was set, the channel was dilated one by one through the metal coaxial dilator to F 21, F 24 nephroscope short sheath was placed, the dilator was removed, the percutaneous nephroscope channel was constructed, the corresponding film sheath was placed, the nephroscope and lithotripsy device was placed, the renal calculi through a clear imaging system was identified, the hydraulic perfusion pump flow was adjusted to 300∼400 L/min, the upper limit of pressure is 200∼300 mmHg, pneumatic ballistic channel was implemented; the larger broken calculi was removed through the ureteral forceps, the small calculi was washed through the perfusion pump and retrograde catheter, lithotripsy was completed, the normal saline was inserted, the lithotripsy was removed, the lithotripsy sheath was inserted again, and the lithotripsy sheath was removed, remove the lithotripsy sheath, remove the lithotripsy, remove the lithotripsy sheath, remove the lithotripsy sheath, remove the lithotripsy, remove the lithotripsy Routine hold of double-J tube.

For the patients in the study group, ercutaneous nephrolithotomy combined with needle nephrolithotomy was performed. First, the standard channel was constructed. The specific measures were the same as the control group. After the completion, lithotripsy was performed by ultrasonic lithotripter. The lithotripsy was crushed into small pieces. The large stones were removed by lavage fluid and stone extraction forceps. With the assistance of B ultrasound, needle nephrolithotomy was performed and inserted into the calyces that were difficult to be touched by standard channel PCNL. The stones were broken by a titanium laser fiber (200 um) and washed out by water. No double-J tube was required to be shelved.

### 2.3. Outcome Measures

(1) The perioperative conditions of the two groups were statistically analyzed, including the length of operation, intraoperative blood loss, stone clearance rate, length of hospital stay, and degree of pain, and the degree of pain was assessed according to the VAS scale, with a total of 10 points, and the lower the score, the better. (2) The levels of renal function (blood urea nitrogen (BUN), serum creatinine (Scr), and cystatin (C) were measured before and 1 d after operation in both groups. (3) The levels of inflammatory factors (C-reactive protein (CRP), procalcitonin (PCT)) before surgery and 1 d after surgery were counted in both the groups. (4) The incidence of complications in the two groups was counted.

### 2.4. Statistical Methods

The data were analyzed by SPSS 22.0 (IBM SPSS Statistics, USA), the data were expressed as mean ± standard deviation (SD). The differences were determined by *t*-test. The two-sided*P* < 0.05 indicated statistically significant differences.

## 3. Results

### 3.1. Perioperative Conditions

There was no significant difference in stone clearance rate between the study group (95.45%) and the control group (90.91%) (*P* > 0.05). The study group was shorter in operation time (42.26 ± 7.03) min, hospital stay (6.09 ± 1.28) d, intraoperative blood loss (12.35 ± 2.43) ml than the control group, and VAS score (2.92 ± 0.96) points than the control group (*P* < 0.05, Table 1).

### 3.2. Renal Function Indicators

There was no significant difference in BUN (6.06 ± 1.45) mmol/L, Scr (75.54 ± 8.48) *μ*mol/L, and CysC (490.11 ± 20.37) *μ*g/L between the study group and the control group before operation (*P* > 0.05). The serum levels of Scr, BUN, and CysC in the two groups at 1 d after operation were higher than those before operation (*P* < 0.05), but BUN (7.51 ± 1.14) mmol/L, Scr (84.68 ± 10.68) *μ*mol/L, and CysC (585.16 ± 32.19) *μ*g/L in the study group were lower than those in the control group (*P* < 0.05), see Table 2.

### 3.3. Inflammatory Factors

There was no significant difference in CRP (17.65 ± 9.24) mg/L and PCT (0.43 ± 0.15) ng/L between the study group and the control group before operation (*P* > 0.05). One day after operation, CRP and PCT in the two groups were higher than those before operation (*P* < 0.05), but CRP (26.69 ± 10.04) mg/L and PCT (0.66 ± 0.17) ng/L in the study group were lower than those in the control group (*P* < 0.05), see Table 3.

### 3.4. Complications

The incidence of complications in the study group (4.55%) was lower than that in control group (18.18%) (*P* < 0.05), see Table 4.

## 4. Discussion

Because complex renal calculi have complex distribution, irregular shape, and large stone diameter, they are easy to cause urinary tract obstruction, infection, and other related complications, causing renal failure, kidney injury, etc., which are a great threat to the life and health of patients [10, 11]. Traditional open surgery requires incision of the renal parenchyma, which is easy to cause serious trauma, has a high incidence of postoperative complications, and is easy to residual stones, so the overall effect is difficult to achieve clinical expectations [12, 13]. Therefore, how to safely and effectively treat complex renal calculi is still a research hotspot.

With the improvement of medical technology, PCNL has gradually become the main treatment for renal calculi, with less trauma and higher safety. However, staged and multichannel surgery is usually required for complex renal calculi to achieve ideal results, but it will increase the medical costs and surgical risks to varying degrees [14–16]. The study pointed out that with the continuous improvement of endoscopic technology, the concept of needle-like nephroscope was developed in clinical practice combined with early ultrasound-assisted puncture needle puncture of parallel calyceal stones and pushing them to the renal pelvis to perform nephroscopic lithotripsy, so as to prevent redilatation and reduce the number of percutaneous renal channels. It can perform direct powdered lithotripsy through laser after successful puncture of the target calyceal calyx without reconstructing the skin renal channel, which can improve the success rate of stone lithotripsy and has a higher safety [17, 18]. At the same time, the treatment procedure was assisted by needle nephroscope, and the stones could be rapidly discharged by high-pressure lavage during the implementation of superior lithotripsy, without the influence of ureteral factors, and the stone clearance effect was satisfactory [19].

The results of this study showed that there was no significant difference in stone clearance rate between the study group and the control group, but other perioperative-related indicators and renal function-related indicators were superior to the control group, and the incidence rate of complications (4.55%) was lower than the control group (18.18%) (*P* < 0.05), indicating that percutaneous nephrolithotomy combined with needle nephrolithotomy has high application value in complex renal calculi, can reduce surgical trauma, help ensure renal function, and the inflammatory response caused by surgical invasive treatment is mild, the incidence rate of postoperative complications is low, and the safety is guaranteed. The main reasons for this analysis are as follows: in needle nephrolithotomy, the diameter of visual fiber is only 0.7 mm, which can transmit high-definition images in real time and clearly, assist physicians to implement relevant treatment operations, try to avoid blood vessels and prevent damage, and break stones through titanium laser during lithotripsy, which can improve the accuracy of surgical treatment and reduce body damage. At the same time, titanium laser is a solid pulse laser, which can produce photothermal effect during application and trigger the thermochemical reaction of stones, thus breaking and clearing stones, and the penetration depth of titanium laser tissue is small, usually no more than 0.5 mm, without obvious side damage to the tissue, ensuring the safety. In addition, not indwelling a double-J tube after surgery can also prevent infection, bleeding, and other related complications caused by the second extubation, in order to reduce the degree of pain and shorten the time of postoperative physical function rehabilitation.

PCT and CRP are commonly used indicators for clinical evaluation of inflammatory response, and their serum content is low under normal physiological conditions, but if the body is injured, it will be abnormally increased, so they can be used to assess the degree of surgical trauma. The results of this study showed that the serum PCT and CRP levels in the study group were lower than those in the control group at 1 d after operation (*P* < 0.05), and it was further confirmed from a microscopic point of view that the combination of percutaneous nephrolithotomy and needle nephrolithotomy for complex renal calculi was feasible and effective, with less trauma, which could reduce the degree of inflammatory response caused by surgical invasive treatment procedures. The main reasons for this analysis are as follows: accurate localization of stone location during surgery is an important prerequisite to ensure the pertinence and effectiveness of treatment. Conventional PCNL requires substantial swing to find stones, which easily produces different degrees of mechanical damage to peripheral organs and blood vessels. Needle nephroscope is small in size, light in weight, and can locate the stone location without substantial swing, so as to effectively reduce the damage to the patient's kidney and reduce the degree of stress response.

In summary, percutaneous nephrolithotomy combined with needle nephrolithotomy is effective in the treatment of complex renal calculi, which can reduce the damage to the body and renal function, with less inflammatory reactions caused by surgery, and a lower incidence of complications, with safety.

## Figures and Tables

**Table 1:** Comparison of perioperative conditions between the two groups.

Group	Number of cases	Procedure duration (min)	Intraoperative blood loss (ml)	Stone clearance (n (%))	Length of stay (d)	VAS (points)
Study group	44	42.26 ± 7.03	12.35 ± 2.43	42 (95.45)	6.09 ± 1.28	2.92 ± 0.96
Control group	44	61.38 ± 10.35	39.97 ± 8.91	40 (90.91)	9.71 ± 3.44	3.87 ± 1.05
*T*/*χ*^2^ value		10.137	19.838	0.179	6.542	4.429
*P* value		<0.001	<0.001	0.672	<0.001	<0.001

**Table 2:** Comparison of renal function indicators between the two groups.

Time	Group	Number of cases	BUN (mmol/L)	Scr (*μ*mol/L)	CysC (*μ*g/L)
Before surgery	Study group	44	6.06 ± 1.45	75.54 ± 8.48	490.11 ± 20.37
	Control group	44	6.42 ± 1.71	72.77 ± 9.09	485.88 ± 22.65
	*T* value		1.065	1.478	0.921
	*P* value		0.290	0.143	0.360

1 d after surgery	Study group	44	7.51 ± 1.14	84.68 ± 10.68	585.16 ± 32.19
	Control group	44	8.78 ± 1.65	93.15 ± 11.79	659.13 ± 38.38
	*T* value		4.201	3.532	9.795
	*P* value		<0.001	0.001	<0.001

**Table 3:** Comparison of inflammatory factors between the two groups.

Time	Group	Number of cases	CRP (mg/L)	PCT (ng/L)
Before surgery	Study group	44	17.65 ± 9.24	0.43 ± 0.15
	Control group	44	19.04 ± 8.78	0.41 ± 0.16
	*T* value		0.723	0.605
	*P* value		0.471	0.547

1 d after surgery	Study group	44	26.69 ± 10.04	0.66 ± 0.17
	Control group	44	35.77 ± 11.38	0.87 ± 0.20
	*T* value		3.969	5.307
	*P* value		<0.001	<0.001

**Table 4:** Comparison of complications between the two groups [n (%)].

Group	Number of cases	Fever	Urine leakage	Hemorrhage	Organ damage	Total occurrence
Study group	44	1 (2.27)	1 (2.27)	0 (0.00)	0 (0.00)	2 (4.55)
Control group	44	3 (6.82)	2 (4.55)	2 (4.55)	1 (2.27)	8 (18.18)
Χ^*2*^ value						4.062
*P* value						0.044

## Data Availability

Data will be available from the corresponding author under reasonable requests.
